This article has been retracted.

# MicroRNA-454 regulates stromal cell derived factor-1 in the control of the growth of pancreatic ductal adenocarcinoma

**DOI:** 10.1038/srep22793

**Published:** 2016-03-15

**Authors:** Yue Fan, Li-Li Xu, Chen-Ye Shi, Wei Wei, Dan-Song Wang, Ding-Fang Cai

**Affiliations:** 1 Department of Integrated TCM & Western Medicine, Zhongshan Hospital, Fudan University, Shanghai 200032, China; 2 Department of General Surgery, Zhongshan Hospital, Fudan University, Shanghai 200032, China; 3 Shanghai Institutes for Biological Sciences, Chinese Academy of Sciences, Institute for Nutritional Sciences, Shanghai 200032, China

## Abstract

Pancreatic ductal adenocarcinoma (PDAC) is a highly malignant carcinoma with an extremely high lethality. We recently reported that hypoxia-inducible factor 1 (HIF-1) targets quiescin sulfhydryl oxidase 1 to facilitate PDAC cell growth and invasion. Here, we analyzed the control of another HIF-1 target, stromal cell derived factor-1 (SDF-1), in PDAC cells. We detected significantly more CD68+ macrophages in the PDAC, compared to normal human pancreas (NT). Since macrophages are recruited to the tissue through their expression of CXCR4 in response to SDF-1, we thus examined the SDF-1 levels in the PDAC specimens. Surprisingly, the SDF-1 protein but not mRNA significantly increased in PDAC, compared to NT. Moreover, a SDF-1-targeting microRNA, miR-454, was found to decrease in PDAC. Promoter luciferase assay confirmed that bindings of miR-454 to 3′-UTR of SDF-1 mRNAs inhibited SDF-1 protein translation. Co-culture of bone marrow derived macrophages and miR-454-modified PDAC cells in a transwell migration experiment showed that macrophages migrated less towards miR-454-overexpressing PDAC cells, and migrated more towards miR-454-depleted cells. Implanted miR-454-depleted PDAC cells grew significantly faster than control, while implanted miR-454-overexpressing PDAC cells grew significantly slower than control. Together, our data suggest that miR-454 may regulate SDF-1 in the control of the growth of PDAC.

Pancreatic ductal adenocarcinoma (PDAC) is one of the most lethal cancers with a 5-year survival rate as low as 5%^1^,^2^. Hence, elucidation of the mechanisms underlying the growth and invasion of PDAC is extremely important for developing novel therapeutic approaches^3^,^4^,^5^,^6^.

The role of microRNAs (miRNAs) in the carcinogenesis has been extensively examined in the past decade. MiRNAs are a class of small, non-coding RNAs of around 20 nucleotides that regulate various biological processes, including tumorigenesis^3^,^7^,^8^,^9^,^10^,^11^,^12^,^13^. Bioinformatics approaches together with functional analyses have predicted one-third of all mammalian genes to be targeted by miRNAs, which mainly regulate protein translation through their base-pairing with the three prime untranslated region (3′-UTR) of the target mRNA^14^,^15^,^16^. Previous studies have shown that microRNAs (miRNAs) play critical roles in the carcinogenesis of PDAC^3^,^17^,^18^,^19^.

Hypoxia is a fundamental biological phenomenon that regulates the development and aggressiveness of many cancers including PDAC^20^,^21^,^22^. The homeostatic responses to hypoxia are greatly governed by the transcription factor hypoxia-inducible factor 1 (HIF-1), which plays pivotal roles in tumorigenesis^22^,^23^,^24^. HIF-1 exerts it functions through many downstream factors. Recently, we showed that HIF-1 targeted quiescin sulfhydryl oxidase 1 (QSOX1) to facilitate pancreatic cancer cell growth and invasion^25^. Stromal cell-derived factor-1 (SDF-1 or CXCL12) is another important downstream target of HIF-1. SDF-1 and its receptor CXCR4 are expressed in complementary patterns during embryonic organogenesis, inflammatory responses and tissue repair^26^,^27^,^28^. Previous studies have demonstrated that HIF-1 is a direct regulator for SDF-1^29^,^30^,^31^,^32^, and the regulatory axis of SDF-1/CXCR4 is important for recruitment of CXCR4+ monocyte/macrophage into the inflammatory sites that are rich for SDF-1^33^,^34^,^35^,^36^. However, the regulation of SDF-1 or CXCL12) by miRNAs has not been analyzed in the carcinogenesis of PDAC.

In the current study, we analyzed the control of SDF-1 in PDAC cells and its effects on tumor growth. We analyzed the regulation of SDF-1 by miR-454 *in vitro* in PDAC cells and the effects of miR-454 on tumor growth *in vivo*.

## Materials and Methods

### Experimental protocol approval

All experimental protocols were approved by the Research Bureau of Zhongshan Hospital from Fudan University. All mouse experiments were approved by the Institutional Animal Care and Use Committee at Zhongshan Hospital from Fudan University (Animal Welfare Assurance). The methods regarding animals were carried out in “accordance” with the approved guidelines.

### Specimens from patients

A total of 32 resected PDAC specimens (PDAC) together with paired adjacent non-cancer pancreatic tissue (NT) were used in this study. All specimens had been histologically and clinically diagnosed at Zhongshan Hospital from Fudan University from 2008 to 2014. For the use of these clinical materials for research purposes, informed consent was obtained from all subjects, and approval from the Institutional Research Ethics Committee were obtained. The methods were carried out in accordance with the approved guidelines.

### Mouse treatments

All mouse experiments were performed according to guide from the Institutional Animal Care and Use Committee at Zhongshan Hospital from Fudan University (Animal Welfare Assurance). Surgeries were performed in accordance with the Principles of Laboratory Care, supervised by a qualified veterinarian. The methods were carried out in accordance with the approved guidelines. All efforts were made to minimize pain and suffering. Female NOD/SCID mice of 12 weeks of age were used in the current study. Five mice were analyzed in each experimental condition.

### Cell line culture and transfection

PANC-1 cell line has been generated from a human carcinoma of the exocrine pancreas in 1975^37^, and was purchased from American Type Culture Collection (ATCC, Rockville, MD, USA). PANC-1 cells were maintained in Dulbecco’s modified Eagle’s medium (DMEM, Invitrogen, Carlsbad, CA, USA) supplemented with 15% fetal bovine serum (FBS; Sigma-Aldrich, St Louis, MO, USA) in a humidified chamber with 5% CO_2_ at 37 °C. MG132 (Sigma-Aldrich) was used in 5 μmol/l in culture to inhibit protein degradation, and the cells were examined 2 hours after MG132 administration. The sequences encoding miR-454, antisense (as)-miR-454, or control null were cloned into pcDNA3.1EGFR vector (Clontech, Mountain View, CA, USA). The transfection was performed with Lipofectamine-2000 (Invitrogen). The success of transfection (more than 95%) was assured by enhanced green fluorescent protein (EGFP) expression of the transfected cells.

### *In vivo* implantation of tumor cells and quantification of tumor size

MiR-454-modified PANC-1 cells (10^6^) were subcutaneously injected under the skin at the back of the NOD/SCID mice. The tumor was allowed to grow for 1 month, dissected out, and then weighed for quantification.

### Quantitative real-time PCR (RT-qPCR)

Total RNA was extracted from tissue, or cells with miRNeasy mini kit (Qiagen, Hilden, Germany). Complementary DNA (cDNA) was randomly primed from 2 μg of total RNA using the Omniscript reverse transcription kit (Qiagen). Quantitative real-time PCR (RT-qPCR) was subsequently performed in triplicate with a 1:4 dilution of cDNA using the Quantitect SyBr green PCR system (Qiagen). All primers were purchased from Qiagen. Data were collected and analyzed using 2-ΔΔCt method for quantification of the relative mRNA expression levels. Values of genes were first normalized against β-actin, and then compared to the experimental control.

### SDF-1 ELISA

The protein was extracted from tissue or cells or conditioned media (secreted protein into the culture media), and then analyzed using SDF1 ELISA kit (R&D Systems, Los Angeles, CA, USA), according to the manufacturer’s instruction.

### Isolation and culture of bone-marrow derived macrophages

Bone-marrow derived macrophages (MΦ) were isolated from a healthy 35-year-old male donor. The marrow was washed 3 times with vehicle solution (PBS containing 20 mmol/l Tris and 100 mmol/l NaCl, pH 7.5). Cells that passed a 40 μm filter were pre-treated with PEcy7-conjugated CD68 antibody (Becton-Dickinson Biosciences, San Jose, CA, USA) and then sorted for positive cells by flow cytometry. The differentiation of bone-marrow-derived monocytes into macrophages was performed as described^38^,^39^. Purified CD68-positive macrophages were cultured in Dulbecco’s Modified Eagle Medium/F12 (DMEM/F12; Invitrogen, St. Louis, MO, USA) supplemented with 10 mmol/l L-glutamine, 100 U/ml penicillin, 100 μg/ml streptomycin and 100 U/ml recombinant CSF (R&D Systems, Los Angeles, CA, USA).

### Fluorescence-activated cell sorting (FACS) for macrophages

Cultured cells or dissociated mouse cancer tissue were detached with 0.25% Trypsine solution (Invitrogen), washed three times with PBS, re-suspended, labeled with PEcy7-conjugated CD68 antibody (Becton-Dickinson Biosciences) for sorting for macrophages. Flow cytometry was performed in a FACSAria flow cytometer (Becton-Dickinson Biosciences). Data were analyzed and quantified using Flowjo software (Flowjo LLC, Ashland, OR, USA).

### Immunohistochemistry

All pancreas samples were fixed in 4% formaldehyde (Sigma-Aldrich) for 6 hours, then cryo-protected in 30% sucrose overnight before freezing. Primary antibody is rabbit polyclonal CD68 antibody (Santa Cruz Biotechnology, Dallas, Texas, USA). The signals were developed by a DAB/ABC assay (DAKO, Carpinteria, CA, USA).

### Luciferase-reporter activity assay

Luciferase-reporters were successfully constructed using molecular cloning technology. The SDF-1 3′-UTR reporter plasmid (SDF-1 3′-UTR) and SDF-1 3′-UTR reporter plasmid with a mutant at the miR-454 binding site (SDF-1 3′-UTR mut) were purchased from Creative Biogene (Shirley, NY, USA). PANC-1 cells were co-transfected with SMAD7 3′-UTR/SMAD7 3′-UTR mut and miR-454/as-miR-454/null by Lipofectamine 2000 (5 × 10^4^ cells per well). Cells were collected 24 hours after transfection for assay using the dual-luciferase reporter assay system gene assay kit (Promega, Beijing, China), according to the manufacturer’s instructions.

### Statistical analysis

All statistical analyses were carried out using the SPSS 18.0 statistical software package. All data were statistically analyzed using one-way ANOVA with a Bonferroni correction, followed by Fisher’s Exact Test. Bivariate correlations were calculated by Spearman’s Rank Correlation Coefficients. All values are depicted as mean ± standard error and are considered significant if p < 0.05.

## Results

### Inverse correlation between SDF-1 and miR-454 in PDAC specimens

We detected more CD68+ macrophages in the PDAC, compared paired normal human pancreas (NT) (Fig. 1A). Since macrophages are well-known to be recruited to the tissue through their expression of CXCR4 in response to SDF-1, we thus examined the SDF-1 levels in 32 PDAC specimens. Surprisingly, the SDF-1 protein by ELISA (Fig. 1B) but not mRNA by RT-qPCR (Fig. 1C) significantly increased in PDAC, compared to NT. These data suggest presence of post-transcriptional control of SDF-1 in PDAC. Since miRNAs are key players that regulate protein translation, we screened the SDF-1-targeting miRNAs, and specifically found that the levels of miR-454 by RT-qPCR significantly decreased in PDAC, compared to NT (Fig. 1D). To test a possible relationship between miR-454 and SDF-1 in PDAC, we performed a correlation test in the 32 PDAC specimens from patients. A strong inverse correlation was detected (Fig. 1Eγ = −070, p < 0.0001, N = 32), suggesting a possible regulatory relationship between miR-454 and SDF-1 in PDAC.

### SDF-1 Protein translation is inhibited by miR-454 in PDAC cells

By bioinformatics analyses, we found that miR-454 bound to 3′-UTR of SDF-1 mRNA at 1466–1472 base site (Fig. 2A). In order to verify that this specific binding is functional, we either overexpressed miR-454, or inhibited miR-454 (by antisense of miR-454; as-miR-454) in a human PDAC cell line, PANC-1. The PANC-1 cells were also transfected with a plasmid carrying a null sequence as a control (null). Co-expression of an EGFP reporter in these plasmids allow purification of transfected cells by flow cytometry. The overexpression or inhibition of miR-454 in PANC-1 cells was confirmed by RT-qPCR (Fig. 2B). MiR-454-modified PANC-1 cells were then transfected with 1 μg plasmids carrying luciferase reporter for 3′-UTR of SDF-1 mRNA. Moreover, null-transfected PANC-1 cells were also transfected with 1 μg plasmids carrying luciferase reporter for 3′-UTR of SDF1 mRNA with one mutate at the miR-454 binding site (mut). The luciferase activities were quantified in miR-454-modified PANC-1 cells, suggesting that miR-454 specifically targets 3′-UTR of SDF-1 mRNA to inhibit its translation (Fig. 2C). Moreover, modification of miR-454 levels in PANC-1 cells did not alter SDF-1 mRNA (Fig. 2D), but significantly altered the cellular (Fig. 2E) and secreted (Fig. 2F) SDF-1 protein. In order to figure out whether miR-454 may affect protein degradation of SDF-1 that contributes to the protein level alteration of SDF-1, we gave these miR-454-modified PANC-1 cells MG132, a specific, potent, reversible and cell-permeable proteasome inhibitor to suppress the cellular protein degradation in miR-454-modified cells. We examined the effects of MG132 on levels of SDF1 and our results showed that SDF-1 degradation seemed not a major contributor to SDF-1 level alteration by miR-454 modulation in PANC-1 cells (Fig. 2D–F).

### MiR-454-depleted PANC-1 cells increase recruitment of macrophages

In order to test whether miR-454 modification may affect the potential of PDAC cells to recruit macrophages through SDF-1, we first isolated bone-marrow-derived macrophages from healthy donor, based on CD68 expression using flow cytometry (Fig. 3A). The isolated CD68+ macrophages were co-cultured with miR-454-modified PANC-1 cells in a transwell system for 48 hours (Fig. 3B). The migrated macrophages into the lower panel were analyzed by flow cytometry based on CD68, since the PANC-1 cells were CD68-negative. We found that macrophages migrated less towards miR-454-overexpressing PDAC cells, and migrated more towards miR-454-depleted cells, shown by representative flow charts (Fig. 3C), and by quantification (Fig. 3D), confirming our hypothesis.

### MiR-454-depleted PANC-1 cells generate bigger tumor *in vivo*

Finally, miR-454-modified PANC-1 cells were implanted into NOD/SCID mice to examine the effects of miR-454 levels on tumor. One month after tumor cell transplantation, the tumor was dissected out, weighed, and then dissociated into single cells for flow cytometry. We found that the CD68+ cell percentage in miR-454-depleted PANC-1-cell-formed tumor was significantly higher than control, while the CD68+ cell percentage in miR-454-overexpressing PANC-1-cell-formed tumor was significantly lower than control, shown by representative flow charts (Fig. 4A), and by quantification (Fig. 4B). In addition, the SDF-1 level in miR-454-depleted PANC-1-cell-formed tumor was significantly higher than control, while the SDF-1 level in miR-454-overexpressing PANC-1-cell-formed tumor was significantly lower than control (Fig. 4C). Moreover, the weight of miR-454-depleted PANC-1-cell-formed tumor was significantly higher than control, while the weight of miR-454-overexpressing PANC-1-cell-formed tumor was significantly lower than control, shown by quantification (Fig. 4D), and by gross images (Fig. 4E). Together, these data suggest that MiR-454-depleted PANC-1 cells generate bigger tumor *in vivo*. Thus, our study suggests that miR-454 may inhibit SDF-1 to promote the growth of PDAC. This model is thus summarized (Fig. 5).

## Discussion

Previous reports have shown that many miRNAs play important roles in the growth and metastasis of PANC cells. Hence, clarification of the aberrant expression of miRNAs in PANC cells may help to determine the mechanisms underlying PANC cell growth and metastases.

We have previously shown that HIF-1 targeted QSOX1 to facilitate pancreatic cancer cell growth and invasion^25^. QSOX1 oxidizes sulfhydryl groups to form disulfide bonds in proteins, and has been found to promote invasion of PDAC cells by activating MMP-2 and MMP-9. We found that both hypoxia and hypoxia mimicking reagent up-regulated the expression of QSOX1 in human PDAC cells. Knockdown of HIF-1 abolished the effects of hypoxia on QSOX1 activation. HIF-1 was found directly bound to two hypoxia-response elements of QSOX1 gene that were required for HIF-1 induced QSOX1 expression. In this study, we analyzed targets of HIF-1 other than QSOX1. We selected SDF-1, since it is a key target of HIF-1^26^,^27^,^28^,^29^,^30^,^31^,^32^, and the regulatory axis of SDF-1/CXCR4 is important for recruitment of CXCR4+ monocyte/macrophage into the SDF-1-rich tumor area.

Indeed, macrophages play an essential role in cancer initiation, formation, progression and migration. Those macrophages that are associated cancer cells are specifically termed as tumor-associated macrophages (TAM), which have been extensively studied for their active and potential participation of the tumorigenesis of various tumors^40^,^41^,^42^,^43^,^44^,^45^,^46^, including PDAC^47^,^48^,^49^,^50^. TAM are well known to express CXCR4, their recruitment, differentiation and polarization as well as their crosstalk with cancer cells depend on the production and secretion of the CXCR4 ligand, SDF-1 by tumor cells. Hence, in this study, we focused on the studies on SDF-1 and TAM in PDAC.

From analyses of PDAC specimens, we found that PDAC contained significantly more CD68+ macrophages, compared to NT, suggesting presence of macrophage recruitment and retention signals in the PDAC tissue. SDF-1 is such a candidate that was later found to significantly increase at protein but not mRNA levels. These data prompted us to examine SDF-1-targeting miRNAs, since miRNAs are one of the key post-transcriptional regulators. We use bioinformatics analyses to screen SDF-1 targeting miRNAs, e.g. miR-301a, miR-301b, miR-3666, miR-130a, miR-130b, miR-4295, miR-454, etc. We found that miR-454 was a SDF-1-targeting miRNA, the levels of which significantly decreased in PDAC. Promoter luciferase assay showed that bindings of miR-454 to 3′-UTR of SDF-1 mRNAs inhibited both cellular and secreted SDF-1, which was further confirmed by analyzing mRNA and protein levels of SDF-1 in miR-454-modified PDAC cells. There seemed to be a significant repression of the mutant UTR in the presence of miR-454. Given that the mutant UTR should not bind miR-454 and yet did not have the same response as the wild type UTR plus antisense, these data may suggest the presence at least one cryptic miR-454 binding site. The large-scale changes in luciferase levels seemed unusual for miRNAs, which may be due to the importance of the binding site of miR-454 on the 3′-UTR of SDF-1 mRNA to its translation. Since there were no difference in the relative changes in cellular and secreted SDF-1 levels in miR-454-modified cells, these data suggest that miR-454 may not affect the secretion level of SDF-1. Since post-transcriptional control of protein levels can be also regulated by protein degradation, we used a potent proteasome inhibitor to suppress the cellular protein degradation in miR-454-modified cells for 2 hours, which did not alter the effects of miR-454 modification on SDF-1 protein. Of note, we have also used this proteasome inhibitor for 4 hours, and got similar results. Thus, the contribution of SDF-1 degradation here seemed very unlikely.

Moreover, we performed a co-culture experiment using bone marrow derived macrophages and miR-454-modified PDAC cells in a transwell migration system. Here, the miR-454-overexpressing PDAC cells produced and secreted significantly less SDF-1, resulting in a decrease in the cross-membrane migration of macrophages, while the miR-454-depleted PDAC cells produced and secreted significantly more SDF-1, resulting in an increase in the cross-membrane migration of macrophages. Finally, we showed that adaptation of TAM in implanted PDAC through miR-454 modification significantly affected cancer cell growth *in vivo*. These data were expected, since TAM produce trophic factors to augment cancer cell proliferation, growth, invasion and survival. We did not analyze macrophage polarization in the current study. However, we think that it is an important question to be answered in future studies.

Previous studies have shown different roles of CXCR4 and miR-454 in various cancers. For example, CXCR4 can act as a tumor suppressor in pancreatic cancer^51^. Additionally, miR-454 has been described as an oncogene^52^,^53^ or tumor suppressor^54^,^55^. These studies suggest that the role of CXCR4 and miR-454 in tumorigenesis may be cancer-specific, which may result from the different levels of their different regulators or targets in various cancers.

Our data were basically achieved from clinical samples and a PANC cell line, while the mechanism parts have been mainly done with the cell line. Validation of these findings using primary PDAC cells may be applied in future. Also, the roles of miR-454/SDF-1 were not completely analyzed in the current study, since there are cell types other than macrophages that may be also affected. For example, the involvement of mesenchymal cells inside and in the periphery of tumor tissue may be studied in future studies, since there are evidence that mesenchymal cells are also regulated SDF-1. For our *in vivo* study, subcutaneous tumor model is not the best model, since tumor microenvironment is crucial to pancreatic cancer. In future, KRAS-mutate pancreatic cancer model may be examined to validate the results in the current study. To summarize, the findings in the current study highlight a role of miR-454/SDF-1 in regulation of TAM in PANC, which may be important for PDAC cell growth.

## Additional Information

**How to cite this article**: Fan, Y. *et al.* MicroRNA-454 regulates stromal cell derived factor-1 in the control of the growth of pancreatic ductal adenocarcinoma. *Sci. Rep.* **6**, 22793; doi: 10.1038/srep22793 (2016).

## Figures and Tables

**Figure 1:** Inverse correlation between SDF-1 and miR-454 in PDAC specimens. A total of 32 resected PDAC specimens (PDAC) together with paired adjacent non-cancer pancreatic tissue (NT) were used in this study. (**A**) Immunostaining for CD68 in the PDAC and NT. (**B,C**) SDF-1 protein levels by ELISA (**B**), and mRNA levels by RT-qPCR (**C**) in PDAC, compared to NT. (**D**) Levels of miR-454 in PDAC by RT-qPCR, compared to NT. (**E**). A correlation test between SDF-1 and miR-454 in the 32 PDAC specimens from patients. *p < 0.05. NS: non-significant. N = 32. Scale bars are 50 μm.

**Figure 2:** SDF-1 Protein translation is inhibited by miR-454 in PDAC cells. (**A**) Bioinformatics analyses showed that miR-454 bound to 3′-UTR of SDF-1 mRNA at 1466–1472 base site. (**B–D**) We either overexpressed miR-454, or inhibited miR-454 (by antisense of miR-454; as-miR-454) in a human PDAC cell line, PANC-1. The PANC-1 cells were also transfected with a plasmid carrying a null sequence as a control (null). (**B**) RT-qPCR for miR-454. (**C**) MiR-454-modified PANC-1 cells were transfected with 1 μg plasmids carrying luciferase reporter for 3′-UTR of SDF-1 mRNA. Moreover, null-transfected PANC-1 cells were also transfected with 1 μg plasmids carrying luciferase reporter for 3′-UTR of SDF1 mRNA with one mutate at the miR-454 binding site (mut). The luciferase activities were quantified. (**D–F**) SDF-1 mRNA (**D**), cellular protein (**E**) and secreted protein (in the culture media as conditioned media, (**F**) in miR-454-modified PANC-1 cells. *p < 0.05. NS: non-significant. N = 5.

**Figure 3:** MiR-454-depleted PANC-1 cells increase recruitment of macrophages. (**A**) Bone-marrow-derived macrophages were isolated from healthy donor, based on CD68 expression using flow cytometry. (**B**) The isolated CD68+ macrophages were co-cultured with miR-454-modified PANC-1 cells in a transwell system for 48 hours. (**C–D**) The migrated macrophages into the lower panel were analyzed by flow cytometry based on CD68, shown by representative flow charts (**C**), and by quantification (**D**). *p < 0.05. N = 5.

**Figure 4:** MiR-454-depleted PANC-1 cells generate bigger tumor *in vivo*. MiR-454-modified PANC-1 cells were implanted into NOD/SCID mice to examine the effects of miR-454 levels on tumor growth. One month after tumor cell transplantation, the tumor was dissected out, weighed, and then dissociated into single cells for flow cytometry. (**A,B**) CD68+ cell percentage from implanted tumor by flow cytometry, shown by representative flow charts (**A**), and by quantification (**B**). (**C**) SDF-1 levels in tumor. (**D,E**) The weight of the implanted tumor (N = 5), shown by quantification (**D**), and by gross images (**E**). *p < 0.05. N = 5.

**Figure 5:** Schematic of the model. MiR-454 may regulate SDF-1 in the control of the growth of PDAC cells.
